The article "Analysis of the Prevalence, Secretion and Function of a Cell Cycle-Inhibiting Factor in the Melioidosis Pathogen Burkholderia pseudomallei" was retracted in 2023. Reasons: concerns about the data; concerns about the results or conclusions.

# Analysis of the Prevalence, Secretion and Function of a Cell Cycle-Inhibiting Factor in the Melioidosis Pathogen *Burkholderia pseudomallei*

**DOI:** 10.1371/journal.pone.0096298

**Published:** 2014-05-08

**Authors:** Pornpan Pumirat, Charles Vander Broek, Niramol Juntawieng, Veerachat Muangsombut, Pattarachai Kiratisin, Kovit Pattanapanyasat, Joanne M. Stevens, Mark P. Stevens, Sunee Korbsrisate

**Affiliations:** 1 Department of Microbiology and Immunology, Faculty of Tropical Medicine, Mahidol University, Bangkok, Thailand; 2 Department of Immunology, Faculty of Medicine Siriraj Hospital, Mahidol University, Bangkok, Thailand; 3 The Roslin Institute and Royal (Dick) School of Veterinary Studies, University of Edinburgh, Midlothian, United Kingdom; 4 Department of Microbiology, Faculty of Medicine Siriraj Hospital, Mahidol University, Bangkok, Thailand; 5 Center of Excellence for Flow Cytometry, Faculty of Medicine Siriraj Hospital, Mahidol University, Bangkok, Thailand; Centre National de la Recherche Scientifique, Aix-Marseille Université, France

## Abstract

Enteropathogenic and enterohaemorrhagic *Escherichia coli* express a cell cycle-inhibiting factor (Cif), that is injected into host cells via a Type III secretion system (T3SS) leading to arrest of cell division, delayed apoptosis and cytoskeletal rearrangements. A homologue of Cif has been identified in *Burkholderia pseudomallei* (CHBP; Cif homologue in *B. pseudomallei*; BPSS1385), which shares catalytic activity, but its prevalence, secretion and function are ill-defined. Among 43 available *B. pseudomallei* genome sequences, 33 genomes (76.7%) harbor the gene encoding CHBP. Western blot analysis using antiserum raised to a synthetic CHBP peptide detected CHBP in 46.6% (7/15) of clinical *B. pseudomallei* isolates from the endemic area. Secretion of CHBP into bacterial culture supernatant could not be detected under conditions where a known effector (BopE) was secreted in a manner dependent on the Bsa T3SS. In contrast, CHBP could be detected in U937 cells infected with *B. pseudomallei* by immunofluorescence microscopy and Western blotting in a manner dependent on *bsaQ*. Unlike *E. coli* Cif, CHBP was localized within the cytoplasm of *B. pseudomallei*-infected cells. A *B. pseudomallei chbP* insertion mutant showed a significant reduction in cytotoxicity and plaque formation compared to the wild-type strain that could be restored by plasmid-mediated *trans*-complementation. However, there was no defect in actin-based motility or multinucleated giant cell formation by the *chbP* mutant. The data suggest that the level or timing of CHBP secretion differs from a known Bsa-secreted effector and that CHBP is required for selected virulence-associated phenotypes *in vitro*.

The article "Analysis of the Prevalence, Secretion and Function of a Cell Cycle-Inhibiting Factor in the Melioidosis Pathogen Burkholderia pseudomallei" was retracted in 2023. Reasons: concerns about the data; concerns about the results or conclusions.

## Introduction

*Burkholderia pseudomallei* is a facultative intracellular pathogen that causes melioidosis, a severe invasive disease of humans that may involve subacute and latent phases. The basis of entry and persistence of *B. pseudomallei* in host cells is ill-defined, but the *bsa*-encoded Inv/Mxi-Spa-like Type III secretion system (T3SS-3) has been identified as a key virulence factor [1], [2]. T3SSs are nano-machines that inject bacterial effector proteins directly into host cells in order to subvert host cellular processes [3]. Only a small number of effectors have been confirmed to be substrates of the Bsa T3SS in *B. pseudomallei*, including BopC [4] and the guanine nucleotide exchange factor BopE [5]. A further candidate effector (BopA) was demonstrated to be Type III secreted in a surrogate bacterial host [6] and to interfere with LC3-associated phagocytosis [7]. A homologue of an *E. coli* Type III secreted effector termed Cif (cycle-inhibiting factor) was identified in *B. pseudomallei* and exhibits 21% amino acid identity and 40% similarity [8], but no evidence has yet been presented that it is secreted via the Bsa apparatus or that it influences pathogenesis during melioidosis.

In a subset of enteropathogenic and enterohaemorrhagic *Escherichia coli* (EPEC and EHEC), Cif is an effector of the locus of enterocyte effacement (LEE)-encoded T3SS [8], [9] and belongs to the cyclomodulin family of proteins that interfere with the eukaryotic cell cycle [10]. Upon contact with epithelial cells, the bacteria inject this protein into the host cell where it induces cell enlargement, arrests the cell cycle G1/S and G2/M transitions, disrupts the actin network, delays cell death and triggers macrophage-specific apoptosis [8], [11]–[13]. Recently, Cif was reported to act by deamidation of ubiquitin or the ubiquitin-like protein NEDD8 that regulates Cullin-RING-ubiquitin ligase (CRL) complexes [14]–[18]. The homologues of *E. coli* Cif in other bacterial pathogens of invertebrates and mammals have been described, including *B. pseudomallei* [15], [17], [19], [20], *Yersinia pseudotuberculosis* [14], [19], *Photorhabdus luminescens* [19]–[21] and *Photorhabdus asymbiotica* [19].

Jubilin et al [19] demonstrated that treatment of HeLa cells with the purified Cif homologue in *B. pseudomallei* (CHBP) mixed with BioPORTER reagent induced cell enlargement, cell cycle arrest at G2 phase and stress fiber formation in an identical manner to that of *E. coli* Cif. Analysis of the crystal structures of CHBP revealed that it possesses a papain-like fold with a Cys-His-Gln catalytic triad similar to *E. coli* Cif [20], [22]. In addition, a recent study showed that CHBP is recognized by melioidosis patient sera [23] indicating that it is expressed *in vivo* and may play a role in pathogenesis.

The article "Analysis of the Prevalence, Secretion and Function of a Cell Cycle-Inhibiting Factor in the Melioidosis Pathogen Burkholderia pseudomallei" was retracted in 2023. Reasons: concerns about the data; concerns about the results or conclusions.

In this study, we investigated the prevalence of CHBP in *B. pseudomallei* strains by genome sequence analysis and by using an antibody raised against a CHBP synthetic peptide to detect the protein in clinical isolates of *B. pseudomallei*. Whilst it is assumed that Cif family members are Type III secreted, no evidence has yet been presented that CHBP is secreted through the Bsa apparatus. We therefore explored whether CHBP is secreted via the Bsa T3SS and evaluated phenotypes of a *B. pseudomallei chbP* mutant and *trans*-complemented strains in a variety of cell culture infection assays.

## Materials and Methods

### Bacterial Strains, Cell Lines and Culture Conditions

The prototype genome-sequenced *B. pseudomallei* strain K96243, *bsaQ* mutant [24] and 14 clinical isolates [25] were routinely maintained in Luria-Bertani (LB) broth or agar (Hardy Diagnostic, USA) containing 40 µg/ml chloramphenicol where needed (*bsaQ*). All cultures were grown at 37°C. Cell lines used in this study including HeLa (human cervical carcinoma), J774A.1 (murine macrophage-like cell) and U937 (human monocyte cell) were obtained from the American Type Culture Collection (ATCC, Manasssas, VA). HeLa, J774.1 and U937 cell lines were routinely maintained in Dulbecco's modified Eagle medium (DMEM) supplemented with 10% (v/v) heat-inactivated fetal bovine serum (FBS). All cells were cultured in a 5% CO_2_ atmosphere at 37°C in a humidified incubator.

### Bioinformatic Analysis of CHBP

The 43 full or partial *B. pseudomallei* genome sequences available at the time of writing were interrogated using the K96243 CHBP protein sequence (accession number NC_006351.1) using a Basic Local Sequence Alignment Tool (tBLASTn) to determine prevalence and sequence conservation. All CHBP amino acid sequences were aligned using Clustal W to identify regions of homology or divergence.

### Construction of *B. pseudomallei chbP* Insertion Mutant and *trans*-complemented Strains

A *B. pseudomallei chbP (bpss1385)* mutant was created by insertion of a plasmid with a conditional origin of replication and chloramphenicol resistance gene into the *chbP* gene on chromosome 2 of strain K92643. A 316 bp internal fragment of *B. pseudomallei chbP* (corresponding to nucleotide positions 183–498) was amplified using primers Cif-f (5′-CTCGGA TCCGAGTTTGAAGATGTTGTTG-3′) and Cif-r (5′-CACTCTAGAAACTGGCG AAAATCCTATG-3′) and the product was cloned into the suicide vector pKNOCK-Cm [26]. The recombinant plasmid pKNOCK-*chbP* was transformed into *E. coli* S17–1λ*pir* [27] and mobilized into *B. pseudomallei* K96243 by conjugation and recipients selected by plating on agar supplemented with 40 µg/ml chloramphenicol and 30 µg/ml kanamycin. The resulting *B. pseudomallei chbP*::pKNOCK mutant was verified by polymerase chain reaction (PCR) using the primer pairs KNOCK1/Cif-R (5′-CACTTAACGGCTG ACATGG-3′/5′-CCGACTAGTACATCTGCTGCGGTCTCAC-3′; product size of 935 bp) and KNOCK2/Cif-F (5′-GTAGCACCAGGCGTTTAA-3′/5′-CCGCT CGAGATGCATCATCATCATCATCATCTACTATTGTTGGAGCACG-3′; product size of 1,584 bp), and by Southern blot analysis using genomic DNA double digested with *Apa*I/*Sma*I enzymes and a *chbP*-specific probe amplified by the Cif-f and Cif-r primers.

The article "Analysis of the Prevalence, Secretion and Function of a Cell Cycle-Inhibiting Factor in the Melioidosis Pathogen Burkholderia pseudomallei" was retracted in 2023. Reasons: concerns about the data; concerns about the results or conclusions.

For complementation studies, the *chbP* open-reading frame was amplified from *B. pseudomallei* K96243 genomic DNA using primers BpsCifTEM (5′-ATATATGAGCTCCAGACAATCTGTGTGGG-3′) and BpsCif6His (5′-ATATATAGATCTCTAGTGGTGGTGGTGGTGGTGGCCAAG GCCGACGACGTATTG-3′). The amplified DNA fragment was cloned into the IPTG-inducible broad host range vector pME6032 [28], generating pCHBP. This plasmid was delivered into the *B. pseudomallei chbP* mutant by electroporation to produce the *B. pseudomallei chbP*/pCHBP strain, which was confirmed by plasmid DNA extraction and sequencing.

### Generation of a CHBP-specific Antibody and Western Blot Analysis

A polyclonal rabbit antiserum against CHBP was generated by Cambridge Research Biochemicals (Cleveland, UK) by immunization with the synthetic peptide ASHEYDFRQFQRNAQ. Specificity of the purified IgG was confirmed by Western blotting of lysates prepared from wild-type *B. pseudomallei* and *chbP* insertion mutant strains. To detect secretion of CHBP in culture supernatants, overnight cultures of *B. pseudomallei* strains were sub-cultured into LB broth or serum-free DMEM with or without induction with 10 mM IPTG where appropriate and incubated at 37°C for 6 h. After centrifugation, *B. pseudomallei* cell pellets were lysed with B-PER II Reagent (Pierce, Rockford, USA) to release intracellular proteins whereas bacterial cell culture supernatant was filtered through 0.22 µM low protein-binding membranes before protein precipitation using a final concentration of 50% (v/v) ethanol. Whole bacterial cell lysates and precipitated secreted proteins were resolved by 12% SDS-polyacrylamide gel electrophoresis (SDS-PAGE) and the proteins were transferred to nitrocellulose membranes (Pierce). The blotted proteins were probed with rabbit BopE-specific [5] or CHBP-specific antibodies at a dilution of 1∶500 for 3 h. Horseradish peroxidase (HRP)-conjugated mouse anti-rabbit IgG (DAKO, USA) at the dilution of 1∶3000 and a chromogenic substrate-3, 3′-diaminobenzidine (DAB; Sigma Chemical Co., USA) were added to detect bound antibodies.

The article "Analysis of the Prevalence, Secretion and Function of a Cell Cycle-Inhibiting Factor in the Melioidosis Pathogen Burkholderia pseudomallei" was retracted in 2023. Reasons: concerns about the data; concerns about the results or conclusions.

For detection of CHBP protein in infected host cells, U937 cells were activated with 20 ng/ml phorbol 12-myristate 13-acetate (PMA; Sigma Chemical Co.) for 48 h in DMEM supplemented with 10% (v/v) FBS then inoculated with *B. pseudomallei* strains at a multiplicity of infection (MOI) of 2 or 100. To induce the expression of CHBP from the pCHBP plasmid in the *trans*-complemented strain, IPTG was added to a final concentration of 10 mM to the culture medium. Two hours after addition of bacterial strains, infected cells were washed with phosphate-buffered saline (PBS) and maintained in media containing 250 µg/ml kanamycin to kill extracellular bacteria for a further 2 h. Media was replaced at 4 h post-infection with fresh medium containing 20 µg/ml kanamycin until 6 h post-infection. Thereafter, the infected cells were washed and lysed with 0.1% (v/v) Triton X-100 in PBS. Protein lysates of infected U937 cells were centrifuged for 1 min at 13,000×g to separate the bacteria and insoluble cytoskeleton of the cells from the cytosolic cell supernatant. Then, the supernatants were resolved by SDS-PAGE, transferred onto nitrocellulose membranes and independently probed with anti-CHBP and anti-BopE antibodies as above. Bound primary antibodies were detected with HRP-conjugated mouse anti-rabbit IgG (DAKO, USA) at a 1∶3000 dilution using SuperSignal West Pico Chemiluminescent substrate (Thermo Scientific Pierce, USA).

### Confocal analysis of CHBP Following Infection

PMA-activated U937 macrophage cells were seeded on 22×22 mm square glass coverslips (Menzel-Glaser, Germany) in 6-well plates (Costar, USA) and incubated at 37°C in a humidified 5% CO_2_ atmosphere. Overnight cultures of *B. pseudomallei* K96243, *chbP* mutant or the *trans*-complemented strain were used to infect U937 cells at a MOI of 2 for 2 h. A 10 mM IPTG (final concentration) was added to the culture medium for induction of CHBP expression from pCHBP. The duration of incubation and procedures for killing of extracellular bacteria were as described above for detection of CHBP in infected cells by Western blotting. At 6 h post-infection cells were washed and fixed with 4% (v/v) paraformaldehyde in PBS. The fixed cells were washed with PBS and permeabilized with 0.5% (v/v) Triton X-100 in PBS for 30 min. Then, 1% (w/v) bovine serum albumin (BSA) in PBS was added and incubated for 30 min at room temperature. Subsequently, the infected cells were stained with 1∶500 of rabbit CHBP-specific antibody at 37°C for 1 h, followed by washing with PBS and bound antibodies were detected with a 1∶1000 goat anti-rabbit antibody-Alexa Fluor^488^ (Molecular Probes, USA) in 1% (w/v) BSA. The staining was observed by confocal laser scanning microscope using a Zeiss LSM 510 META instrument (Carl Zeiss, Germany) and analyzed by DP Manager (version 3.1.1) equipped with LSM (release 3.2) software. Where necessary coverslips were stained for actin filaments using Alexa Fluor^568^-conjugated phalloidin (Molecular Probes) and DNA stained using 4′, 6′ diamidine-2′-phenylindole dihydrochloride (DAPI, Molecular Probes). Bacteria were stained using mouse monoclonal anti-*B*. *pseudomallei* lipopolysaccharide antibody (Camlab, Cambridge, United Kingdom) detected with Alexa Fluor^488^-conjugated anti-mouse Immunoglobulin (Molecular Probes).

The article "Analysis of the Prevalence, Secretion and Function of a Cell Cycle-Inhibiting Factor in the Melioidosis Pathogen Burkholderia pseudomallei" was retracted in 2023. Reasons: concerns about the data; concerns about the results or conclusions.

### Cell Infection Assays

To assay net intracellular replication**,** PMA-activated U937 cells were seeded and infected with *B. pseudomallei* strains at an MOI of 2. After 2 h infection at 37°C, cells were washed with PBS, media was replaced with medium containing 250 µg/ml of kanamycin to kill extracellular bacteria, and incubated for another 2 h. Thereafter, the infected cells were incubated with medium containing 20 µg/ml kanamycin. At 3, 6, 9 and 12 h post-infection, the infected host cells were washed with PBS and lysed with 0.1% (v/v) Triton X-100 in PBS. Viable intracellular bacteria were quantitated by plating serial ten-fold dilutions of lysates on trypticase soy agar and counting colonies after 24–36 h of incubation at 37°C.

Plaque-forming efficiency was evaluated as previously described [29] with some modifications. HeLa cells were infected with *B. pseudomallei* at an MOI of 20 and incubated at 37°C with 5% CO_2_ for 2 h. After 2 h incubation, the infected cell monolayers were washed and replaced with a medium containing kanamycin (250 µg/ml). The plates were incubated at 37°C in a humidified 5% CO_2_ atmosphere for at least a further 16 h. Plaques were stained with 1% (w/v) crystal violet in 20% (v/v) methanol and counted by microscopy. Plaque-forming efficiency was calculated by the following equation: number of plaques/CFU of bacterial added per well.

The efficiency of multinucleated giant cell (MNGC) formation [29] and cell cytotoxicity [30] in monolayers infected with wild-type, the *chbP* mutant and the *trans*-complemented strains of *B. pseudomallei* were assessed as described by Suparak et al [29] and Korbsrisate et al [30].

### Statistical Analysis

All experiments were independently performed a minimum of three times. The significance of differences between groups was assessed using the unpaired *t*-test using GraphPad Prism 6 software (STATCON). P values ≤0.05 were taken to be significant.

The article "Analysis of the Prevalence, Secretion and Function of a Cell Cycle-Inhibiting Factor in the Melioidosis Pathogen Burkholderia pseudomallei" was retracted in 2023. Reasons: concerns about the data; concerns about the results or conclusions.

## Results

### Prevalence and Sequence Diversity of CHBP in *B. pseudomallei*

*B. pseudomallei* K96243 chromosome 2 harbors *bpss1385*, the gene encoding the Cif homologue CHBP, a hypothetical 328 amino acid protein with a predicted molecular weight of 35.8 kDa. To examine the conservation of CHBP among sequenced *B. pseudomallei* strains, 43 available complete or draft *B. pseudomallei* genome sequences were searched for homologues to the CHBP protein of K96243 using tBLASTn and homologous sequences aligned using the ClustalW multiple sequence alignment tool. Of the 43 available genomes, 33 (76.7%) *B. pseudomallei* strains harbored CHBP with >99% amino acid sequence identity to CHBP of *B. pseudomallei* strain K96243. Apart from amino acid differences detected at E32G, T88M, G157R, G223E, G237E and T278M in a small number of strains, the amino acid sequences were remarkably highly conserved, with complete conservation of the predicted catalytic Cys-His-Gln triad [20] (Figure S1). A 1.5 kb deletion of *chbP* (*bpss1385*) between the predicted transposase genes *bpss1384* and *bpss1385a* was detected in the draft genome sequence of the virulent strain 10276 used to identify the *bsa* locus, and was confirmed by PCR with flanking primers (data not shown). The same deletion boundaries were present in all the deposited genome sequences that lack *chbP*, indicating that the gene is likely to be absent in these strains rather than *chbP* sequence reads being absent or not aligned to the scaffold. It is noteworthy that *chbP* homologues were lacking in the related but avirulent species *B. thailandensis* (6 genomes) and the glanders pathogen *B. mallei* (10 genomes). In addition, there was no evidence of any truncations in the *chbP* sequences that may ablate function as described previously from analysis of *E. coli* Cif sequences [8].

Additionally, a selection of *B. pseudomallei* clinical isolates from the endemic area [25] were studied by Western blotting of bacterial cell lysates for CHBP expression using rabbit polyclonal antiserum raised against a CHBP synthetic peptide. Of 15 *B. pseudomallei* isolates, a protein of the expected size of CHBP was detected in 7 (46.6%) samples, whereas 8 samples including the 10276 strain from Bangladesh were negative (data not shown), consistent with the deletion of *chbP* detected in the draft genome sequence and PCR with *chbP*-flanking primers of 10276 genomic DNA.

### Analysis of CHBP Secretion by *B. pseudomallei*

To confirm the specificity of the anti-CHBP antibody and determine if CHBP is secreted, *B. pseudomallei* strains in which *chbP* was inactivated by insertion of the pKNOCK suicide replicon via homologous recombination (*chbP*::pKNOCK) or restored by inducible expression of *chbP* from a plasmid (*chbP*/pCHBP) were constructed and validated by sequencing. Western blot analysis of whole cell extracts of such strains with anti-CHBP detected a protein of the expected size in wild-type K96243, but not the *chbP* insertion mutant, and this was restored by introduction of pCHBP into the mutant (Figure 1). No significant difference in growth of the bacterial strains under the conditions used was detected (data not shown). *B. pseudomallei* Bsa-secreted proteins such as BopE and BipD can be detected in the supernatant of late logarithmic phase LB-grown cultures of wild-type, but not *bsa*-deficient strains [5], [24]. Interestingly, under these conditions, CHBP could not be detected in the supernatant of the cultures that yielded CHBP in the whole cell extract (Figure 1), even though we were able to confirm that the supernatants contained the known Bsa effector BopE by Western blotting using anti-BopE antibody (Figure 1). These data suggest that secretion of CHBP may be regulated in a manner distinct from BopE, though we cannot preclude the possibility that failure to detect CHBP in culture supernatant may reflect low abundance, low antibody affinity or avidity or the insensitivity of the detection system.

The article "Analysis of the Prevalence, Secretion and Function of a Cell Cycle-Inhibiting Factor in the Melioidosis Pathogen Burkholderia pseudomallei" was retracted in 2023. Reasons: concerns about the data; concerns about the results or conclusions.

**Figure 1:** SDS-PAGE and Western blot analysis of CHBP in *B. pseudomallei* K96243 wild-type, *chbP* mutant and *trans*-complemented strains. A) SDS-PAGE. Bacterial lysates and secreted proteins of *B. pseudomallei* K96243, *chbP* mutant or *chbP*/pCHBP strain cultured in LB broth for 6 h were separated by 12% polyacrylamide gel electrophoresis. B) Western blot analysis. The blotted proteins from A) were separately probed with anti-CHBP and anti-BopE antibodies. Molecular mass markers are shown on the left. Lanes 1–3 are bacterial cell lysates and lanes 4–6 are secreted proteins precipitated from culture supernatants.

### CHBP can be Detected in *B. pseudomallei*-infected Cells

Since CHBP could not be detected in *B. pseudomallei* culture supernatants under conditions where BopE was detected, we investigated whether host cell contact may trigger CHBP secretion. U937 macrophage-like cells were separately infected with *B. pseudomallei* K96243, the *chbP* mutant and the *trans*-complemented strain. After 6 h, cells were fixed and stained with rabbit anti-CHBP antibody followed by anti-rabbit Alexa Fluor^488^ conjugate. Confocal micrographs revealed diffuse punctate staining in the cytoplasm of *B. pseudomallei* K96243-infected cells; but with the same conditions for excitation and capture of confocal images, such staining was absent in cells infected with the *chbP* mutant (Figure 2). No differences in intracellular survival of the *B. pseudomallei* K96243 and *chbP* mutant strains were detected over the duration of the assay (Figure S2). The intensity of staining was restored by induction of CHBP expression from a plasmid in the *chbP* mutant (Figure 2). These results indicate that *B. pseudomallei* K96243 is able to secrete CHBP in infected host cells, and that unlike BopE its secretion may require host cell contact.

The article "Analysis of the Prevalence, Secretion and Function of a Cell Cycle-Inhibiting Factor in the Melioidosis Pathogen Burkholderia pseudomallei" was retracted in 2023. Reasons: concerns about the data; concerns about the results or conclusions.

**Figure 2:** Confocal micrographs of CHBP expression and localization in U937 cells infected with *B. pseudomallei*. PMA-activated U937 cells were separately infected with three strains of *B. pseudomallei* (K96243, *chbP* mutant or *chbP*/pCHBP strain). After 6 h, infected cells were fixed, permeabilized andstained using purified rabbit anti-CHBP antibody detected with anti-rabbit Ig-Alexa Fluor^488^ (Molecular Probes). The bottom panel shows the localization of CHBP and the top panel merges this signal with differential interference contrast (DIC) images showing the position of infected cells. Scale bars, 20 µm.

To exclude the possibility that CHBP secretion might be influenced by eukaryotic cell culture medium, bacterial lysates and secreted proteins of *B. pseudomallei* strains cultured in serum-free DMEM were prepared and Western blot analysis of CHBP secretion was performed. CHBP and BopE could not be detected in the supernatants of cultures of the *B. pseudomallei* strains, even though both effector proteins were identified in the bacterial lysates (except from *B. pseudomallei chbP* mutant which does not produce CHBP protein) (Figure S3). This implies that CHBP is secreted in response to host cell infection rather than cues from the culture medium.

The timing of expression and localization of CHBP in infected cells was also followed over time by confocal microscopy. In U937 cells infected with *B. pseudomallei* K96243, staining was consistently detected in the cytoplasm at intervals from 3 to 12 h post-infection (Figure 3), with no obvious concentration in the nucleus as previously reported for *E. coli* Cif over the time intervals tested [19]. Staining could not be detected in the cytosol of U937 cells infected with the *B. pseudomallei chbP* mutant over the same 12 h time course.

**Figure 3:** Confocal micrographs indicating *bsaQ*-dependent secretion of CHBP in U937 cells infected with *B. pseudomallei*. PMA-activated U937 cells were separately infected with *B. pseudomallei* (K96243, *bsaQ* or *chbP* mutant strain). At different time points of infection (3, 6, 9 and 12 h), infected cells were stained using purified rabbit anti-CHBP antibody detected with anti-rabbit Ig-Alexa Fluor^488^ (Molecular Probes). The bottom panel shows the localization of CHBP and the top panel merges this signal with DIC images showing the position of infected cells. Scale bars, 10 µm.

The article "Analysis of the Prevalence, Secretion and Function of a Cell Cycle-Inhibiting Factor in the Melioidosis Pathogen Burkholderia pseudomallei" was retracted in 2023. Reasons: concerns about the data; concerns about the results or conclusions.

The immunofluorescence microscopy data were verified by detection of CHBP protein in infected cells by Western blotting. When using the same MOI and duration of incubation as used for immunofluorescence microscopy CHBP could be detected in lysates of U937 cells infected with the wild-type and *trans*-complemented strains, but not the *chbP* mutant (Figure 4A). BopE could be detected in cells infected with each of the strains, with the exception of the *bsaQ* mutant, and the intensity of signals were increased when an MOI of 100 was used (Figure 4B). The absence of BopE in the lysates of *bsaQ*-infected cells indicates that the signals obtained did not arise from the lysis of bacteria in the samples.

**Figure 4:** SDS-PAGE and Western blot analysis of CHBP in *B. pseudomallei-*infected U937 cells. A) Protein from lysates of U937 cells infected at an MOI of 2 with *B. pseudomallei* K96243, *chbP* mutant, *chbP*/pCHBP strain or *bsaQ* mutant for 3 or 6 h were separated by 12% polyacrylamide gel electrophoresis and blotted with anti-CHBP and anti-BopE antibodies. Molecular mass markers are shown on the left. Panel B shows data from an identical experiment, except using an MOI of 100.

### Secretion of CHBP in Host Cells is Bsa-dependent

As it has been reported that CHBP can be injected by the *E. coli* T3SS in an identical manner to *E. coli* Cif [19], we speculated that CHBP can be secreted via the virulence-associated Bsa T3SS. To investigate this possibility, cells were infected with *B. pseudomallei* wild-type or an isogenic *bsaQ* mutant [24]. The *B. pseudomalle*i *bsaQ* mutant lacks a structural component of T3SS and exhibits a defect in secretion of the known Bsa-secreted proteins BopE and BipD and delayed escape from endosomes [24]. During the 12 h infection time course, the *bsaQ* mutant exhibited comparable intracellular net replication in U937 cells to the *B. pseudomallei* wild-type K96243 strain (Figure S4). Confocal microscopy indicated that the *bsaQ* mutant could not secrete CHBP into the cell cytoplasm even at 12 h post-infection, despite the ability of the *bsaQ* mutant to express the protein as shown in Figure S4. In addition, Western blotting for CHBP in U937 cells infected with the *bsaQ* mutant failed to detect CHBP in cell lysates either at an MOI of 2 (Figure 4A) or 100 (Figure 4B). The data indicate that CHBP secretion in host cells is Bsa-dependent, though further studies are required to determine if this reflects the direct requirement for Bsa to secrete CHBP or the requirement for Bsa-dependent bacterial escape to the cytosol where CHBP may then be secreted.

The article "Analysis of the Prevalence, Secretion and Function of a Cell Cycle-Inhibiting Factor in the Melioidosis Pathogen Burkholderia pseudomallei" was retracted in 2023. Reasons: concerns about the data; concerns about the results or conclusions.

### *B. pseudomallei* CHBP Influences Virulence-associated Interactions with Host Cells

During EPEC and EHEC infections, Cif was initially reported to induce a progressive cytopathic effect involving stress fibre formation, as well as arrest of the cell cycle as detected by a change in DNA content [19]. These phenotypes took several days to fully develop, and it was possible to sterilise the cell cultures of bacteria after a period of T3SS-mediated injection of Cif by antibiotic treatment. We repeatedly attempted to sterilise cell cultures infected with *B. pseudomallei* wild-type and *chbP* mutant strains to investigate effects on the cytoskeleton and cell cycle, but were impeded by the high intrinsic resistance of *B. pseudomallei* to diverse antibiotics and loss of viability of infected host cells at the intervals where phenotypes had previously been detected (data not shown). We were nevertheless able to examine whether CHBP influenced interactions between *B. pseudomallei* and host cells that have been linked to virulence.

The capacity for cell-to-cell spread is an important characteristic of *B. pseudomallei* pathogenesis [31]. The ability of *B. pseudomallei* K96243 and the *chbP* mutant to disseminate from cell-to-cell was evaluated by infection of non-phagocytic HeLa cells. We found that plaque-forming efficiency of *B. pseudomallei chbP* mutant (7.6±3.7×10^−4^ pfu/bacteria) was significantly reduced compared to the wild-type strain (28.7±4.4×10^−4^ pfu/bacteria) (Figure 5A). Moreover, the *B. pseudomallei chbP* mutant consistently produced smaller plaques when compared to the wild-type strain (Figure 5B). Cell-to-cell spreading of the *chbP* mutant was restored by introduction of pCHBP and infection of cells in the presence of inducer.

**Figure 5:** Effect of *chbP* mutation on *B. pseudomallei* plaque formation. A) Plaque-forming efficiency. HeLa cells were infected with *B. pseudomallei* (K96243, *chbP* mutant or *chbP*/pCHBP strain) at an MOI of 20. Plaque-forming efficiency was established following staining of the infected cells with crystal violet. Plaque-forming efficiency at 21 h was calculated by the following equation: number of plaques/CFU of bacteria added per well. Asterisks indicate significant differences (P value <0.05, *t*-test) between groups. Error bars represent standard errors of the means for experiments performed in triplicate. B) Photographs of plaques. Representative images of the infected cell monolayers after infection with *B. pseudomallei* K96243, *chbP* mutant or *chbP*/pCHBP strains for 21 and 24 h. Note the reduced number of plaques and reduced plaque size of the *chbP* mutant.

The article "Analysis of the Prevalence, Secretion and Function of a Cell Cycle-Inhibiting Factor in the Melioidosis Pathogen Burkholderia pseudomallei" was retracted in 2023. Reasons: concerns about the data; concerns about the results or conclusions.

Additionally, we compared the level of host cell damage (cytotoxicity) induced by *B. pseudomallei* wild-type and *chbP* mutant by measuring the LDH release of infected HeLa cells and U937 cells at 6 h post-infection. The *B. pseudomallei chbP* mutant caused a significantly lower level of cytotoxicity compared to the wild-type strain upon infection of HeLa cells (at the MOI of 25, 50 and 100; Figure 6A) and U937 cells (at the MOI of 25 and 50; Figure 6B).

**Figure 6:** Effect of *chbP* mutation on *B. pseudomallei-*induced cytotoxicity. A) HeLa cells and B) U937 cells were infected with *B. pseudomallei* (K96243, *chbP* mutant or *chbP*/pCHBP strain) with a range of MOIs. After 6 h, cytotoxicity was assessed using the CytoTox96 lactate dehydrogenase (LDH)-release kit (Promega). Asterisks indicate significant differences (P value <0.05, *t*-test) between groups. Error bars represent standard errors of the means for experiments performed in triplicate.

## Discussion

Cif is a bacterial cyclomodulin that arrests the cell cycle and modulates multiple cellular processes, as first described during EPEC and EHEC infection of cultured cells [8]. Proteins homologous to *E. coli* Cif have been identified in diverse bacterial pathogens including *Y. pseudotuberculosis*, *P. luminescens*, *P. asymbiotica* and *B. pseudomallei* [19]. Though the subject of intense study at the molecular level; the prevalence, secretion and role in infection of Cif homologues has received little attention. Recently, it has been reported that CHBP is recognized by melioidosis patient sera [23], however its function during interactions between *B. pseudomallei* and host cells is ill-defined.

Analysis of draft or complete *B. pseudomallei* genome sequences available at the time of writing indicated that *chbP* is present in 33 of 43 strains (76.7%), with minimal variation in predicted amino acid sequences and full conservation of the catalytic triad in CHBP-positive strains. A survey of 15 clinical *B. pseudomallei* isolates from the endemic area indicated that approximately half produced CHBP, indicating that CHBP is not an absolute requirement for *B. pseudomallei* to cause melioidosis (or *B. mallei* to cause glanders). Indeed, the *B. pseudomallei* 10276 strain isolated from a human melioidosis patient in Bangladesh is known to be virulent in murine models of melioidosis [32] despite the proven deletion in the *bpss1384*-*bpss1385a* region and absence of CHBP protein by Western blotting with specific antibody. Similarly, Marchès et al [8] reported that *cif* is not universally present in pathogenic EPEC and EHEC, and that some strains encode a truncated variant that is inactive. Variation in the repertoire of Type III secreted effectors is well known and it is possible that CHBP is non-essential for virulence, that functional redundancy may exist, or that presence or absence of Cif is related to subtle differences in virulence. Other cyclomodulins are known in *E. coli* (e.g. cytolethal-distending toxin and cytotoxic necrotizing factor) and it will be of interest to determine if other toxins of this kind exist in pathogenic *Burkholderia*.

The article "Analysis of the Prevalence, Secretion and Function of a Cell Cycle-Inhibiting Factor in the Melioidosis Pathogen Burkholderia pseudomallei" was retracted in 2023. Reasons: concerns about the data; concerns about the results or conclusions.

*B. pseudomallei* is predicted to encode three Type III protein secretion systems and it has yet to be demonstrated that CHBP is secreted by the virulence-associated Bsa apparatus. An antibody raised against a synthetic peptide of CHBP reacted specifically with a 35 kDa protein in whole cell lysates of *B. pseudomallei* K96243 consistent with predictions, but no protein was detected at this position in a lysate of an isogenic *chbP* insertion mutant. Reactivity was restored when cloned *chbP* was introduced into the mutant on an inducible plasmid. In contrast to BopE, which was readily detected in the supernatant of LB-grown *B. pseudomallei* as before [5], we were unable to detect CHBP despite evidence that the protein was present in the whole-cell fraction. Interestingly, we were able to detect CHBP-specific staining in the cytosol of U937 human macrophage cells after infection with *B. pseudomallei* K96243 or the *trans*-complemented strain, but not the *chbP* mutant, suggesting that secretion of CHBP may be activated on host cell contact or induced by an intracellular signal. It is noteworthy that the *P. luminescens* Cif homologue CHPL is secreted into the culture supernatant at a time when the well characterized Type III secreted effector LopT is not [21], even though it has been proposed to be an effector of the T3SS.

Despite the absence of CHBP in the secreted fraction when BopE was detected, appearance of cytosolic CHBP in infected cells was dependent on a functional Bsa system, as it was absent in a *bsaQ* mutant previously reported to be deficient in Type III secretion [4]. Though it is tempting to speculate that the failure of CHBP to appear in lysates of U937 cells infected with the *bsaQ* mutant is evidence that CHBP is secreted via the Bsa apparatus, it should be noted that Bsa is required for the bacteria to escape endosomes. It remains a possibility that CHBP is secreted only once *B. pseudomallei* enters the cytosol in a Bsa-dependent way. To separate these possibilities we repeatedly attempted to detect the Bsa-dependent appearance of CHBP in cells infected with *B. pseudomallei* wild-type and mutant strains in the presence of cytochalasin D to prevent bacterial uptake. By Western blotting we were unable to detect injection of CHBP into cells where *B. pseudomallei* was prevented from uptake (data not shown), though this may reflect low levels of injection or the sensitivity of the detection method,

The cytosolic staining obtained with a CHBP-specific antibody is in contrast to observations with *E. coli* Cif, where ectopic expression leads to accumulation of the protein in the nucleus [16]. CHBP is predicted to act on nuclear targets, but we cannot preclude the possibility that it enters the nucleus at lower levels, or that it may be enriched in the nucleus at time intervals beyond those studied here.

The article "Analysis of the Prevalence, Secretion and Function of a Cell Cycle-Inhibiting Factor in the Melioidosis Pathogen Burkholderia pseudomallei" was retracted in 2023. Reasons: concerns about the data; concerns about the results or conclusions.

*E. coli* Cif induces the accumulation of p21 and p27 that inhibit CDK1-CyclinB and CDK2-CyclinA/E, leading to cell cycle arrest at the G2/M and G1/S transitions [16]. Cui et al [17] demonstrated that this and other activities of Cif require glutamine deamidation of ubiquitin or the ubiquitin-like protein NEDD8 that regulates Cullin-RING ubiquitin ligases. We repeatedly attempted to detect CHBP-dependent inhibition of the cell cycle during *B. pseudomallei* infection as previously demonstrated by *E. coli* Cif by flow cytometric analysis of propidium iodide-stained cells, but were hindered by our inability to completely remove *B. pseudomallei* from the culture system owing to its intrinsic high level of resistance to antibiotics and induction of cell death 24–48 h post-inoculation.

It has been reported that EPEC Cif induces cell damage and apoptosis of IEC-6 intestinal cells in a manner associated with LDH release and caspase-3 activation after infection [12]. Similarly, Cif homologue in *P. luminescens* triggers apoptosis in insect cells, albeit this activity is not associated with virulence in an insect model [21]. Consistent with these findings, the *B. pseudomallei chbP* mutant caused the release of lower levels of LDH in infected HeLa cells compared to the wild-type and complemented strain, despite intracellular net replication occurring at comparable levels (data not shown). *B. pseudomallei* has recently been reported to induce expression of apoptosis-related genes including caspase-3, caspase -8, caspase -9, Bax, and Bcl-2 in macrophages [33], and the role of CHBP in modulation of apoptosis during *B. pseudomallei* infection merits future study, ideally in murine models.

A significant reduction in plaque formation was detected with the *chbP* mutant that could be restored by plasmid-mediated *trans*-complementation. Plaque formation reflects the outcome of multiple processes, including uptake, endosome escape, net intracellular replication and spread to adjacent cells via actin-based motility or cell fusion. While we did not detect a defect in the net intracellular replication (Figure S2), actin tail formation or multinucleated giant cell formation (Figure S5) by the *chbP* mutant over short duration cell-based assays, it is possible that subtle phenotypes are amplified over the longer duration and multiple cycles of infection required to form a plaque. It is noteworthy that despite marked cell-based phenotypes, Cif homologue in *P. luminescens* is not required for full virulence in an insect model [21] and studies in murine melioidosis models are required before the relevance of the activities attributed to CHBP to date can be stated. Nevertheless, our study indicates a requirement for the Bsa apparatus for secretion of CHBP in host cells and indicates that distinct signals may regulate the expression or secretion of Bsa effectors.

The article "Analysis of the Prevalence, Secretion and Function of a Cell Cycle-Inhibiting Factor in the Melioidosis Pathogen Burkholderia pseudomallei" was retracted in 2023. Reasons: concerns about the data; concerns about the results or conclusions.

## Supporting Information

Figure S1 **Sequence diversity of CHBP in sequenced** ***B. pseudomallei*** **genomes.** Prototypic *B. pseudomallei* CHBP sequences were aligned using ClustalW. Note the minor differences in amino acid composition between the proteins (presented in red) and conservation of the predicted catalytic Cys-His-Gln triad (highlighted in yellow) proposed by Crow et al [20].
(TIF)

Figure S2 **SDS-PAGE and Western blot analysis of CHBP in** ***B. pseudomallei*** **K96243, the** ***chbP*** **mutant and the complemented strains grown in DMEM or LB media.** A) *B. pseudomallei* lysates and B) secreted proteins from K96243 wild-type, *chbP* mutant or *chbP*/pCHBP strains cultured in serum-free DMEM medium for 6 h were separated by 12% SDS-PAGE. The blotted proteins were separately probed with anti-CHBP and anti-BopE antibodies. Molecular mass markers are shown on the left of the gel. Bacterial lysate and secreted protein prepared from *B. pseudomallei* K96243 cultured in LB broth were used as the positive controls.
(TIF)

Figure S3 ***B. pseudomallei*** **intracellular survival in U937 cells.** PMA-activated U937 cells were infected with *B. pseudomallei* K96243 wild-type, *bsaQ* or *chbP* mutant strains at an MOI of 2. After 3, 6, 9 and 12 h of infection, infected cells were lysed and the numbers of viable bacteria were enumerated after plating on TSA and incubation at 37°C for 36–48 h.
(TIF)

Figure S4 **SDS-PAGE and Western blot analysis of CHBP expression and secretion in** ***B. pseudomallei*** **K96243 and an isogenic** ***bsaQ*** **mutant.** A) SDS-PAGE. Bacterial lysates and secreted proteins of *B. pseudomallei* K96243 or *bsaQ* mutant strain cultured in LB broth for 6 h were separated by 12% SDS-PAGE. B) Western blot analysis. The blotted proteins from A) were probed with anti-CHBP antibody. Molecular mass markers are shown on the left.
(TIF)

Figure S5 **Effect of** ***chbP*** **mutation on** ***B. pseudomallei*** **intracellular movement and intercellular spreading.** A) Actin tail formation. PMA-activated U937 cells were infected with two strains of *B. pseudomallei* (K96243 or *chbP* mutant strain) at an MOI of 2. After 6 h of infection, infected cells were fixed using 4% paraformaldehyde and actin filaments stained with phalloidin^568^ (red) and bacteria stained with mouse monoclonal anti-*B*. *pseudomallei* lipopolysaccharide antibody detected with anti-mouse Ig-Alexa Fluor^488^ (green). Bar, 10 µm. B) Multinucleated giant cell formation. MNGC formation in J774A.1 murine macrophage cells infected at an MOI of 2 with *B. pseudomallei* (K96243 or *chbP* mutant strain) was studied 6 h post-infection by Giemsa staining of the cell monolayers. The stained cells were examined under a light microscope (OLYMPUS) at a magnification of 20X.
(TIF)
